This article has been retracted.

# Among Live and Dead Bacteria, the Optimization of Sample Collection and Processing Remains Essential in Recovering Gut Microbiota Components

**DOI:** 10.3389/fmicb.2019.01606

**Published:** 2019-07-10

**Authors:** Sara Bellali, Jean-Christophe Lagier, Didier Raoult, Jacques Bou Khalil

**Affiliations:** ^1^IRD, APHM, MEPHI, IHU Méditerranée Infection, Aix Marseille Université, Marseille, France; ^2^IHU Méditerranée Infection, Marseille, France

**Keywords:** culturability, viability, sample processing, protectant medium, microbiota

## Abstract

The human gut microbiota plays an important role in human health. Accessing and culturing the gut microbes remains critical in microbiology. The culturomics approach, combined with sequencing strategies, provides new insights in the study of gut microbiota components. However, we are still far from having described all the microbes. Many factors are involved in recovering as much bacteria as possible. One of the most important factors is sample preparation and conservation. The aim of the present work was to evaluate three different types of stool sample conditioning by mainly studying the effect of atmospheric oxygen on bacterial viability and culturability. Quantitative analysis of fecal samples from eight different healthy individuals was carried out using a culture-independent method (flow cytometry) and a culture-dependent method (plating technique). We found that the cultured bacteria reached a 50% yield when the samples were exposed to oxygen for 120 min without any protectant medium, while the percentage of culturability increased to 67% in the presence of antioxidants. More importantly, when samples were exposed to oxygen for less than 2 min, combined with the work under the anaerobic chamber, no discordance was found between the two counting techniques and the culturability increased to 87%. Our study confirmed the importance of sample conditioning to preserve the bacterial viability in samples, especially for oxygen-sensitive intestinal bacteria.

## Introduction

The human microbiota in general and the gut microbiota in particular remain a clinical research subject of predilection; especially as it plays a key role in health and disease (Sekirov et al., 2010). Scientists are still trying to extensively explore and describe this microbiota, which is the subject of many debates (Eckburg et al., 2005).

Different approaches were used, all with a single objective: to target all microbes. However, all the tested approaches had advantages and drawbacks, leaving a large part of the microbiota unexplored (Lagier et al., 2012a, b; Rinke et al., 2013; Browne et al., 2016). Culturomics, which consists of multiple culture conditions combined with rapid identification of bacteria by MALDI-TOF mass spectrometry, has enabled, through a high isolation rate, the culture of hundreds of new microorganisms that are associated with humans, offering interesting new perspectives into host–bacteria relationships (Lagier et al., 2016, 2018; Bilen et al., 2018). Other recent microbial studies have improved their effectiveness to isolate new microorganisms using YCFA and MPYG (Forster et al., 2019; Zou et al., 2019).

In addition, metagenomics and new generation sequencing strategies capable of recovering DNA and RNA from any sample convinced scientists that they had discovered almost all the bacterial content of our gut microbiota (Almeida et al., 2019; Nayfach et al., 2019; Pasolli et al., 2019). However, many discrepancies have been found, and we are far from having described the whole gut microbiota (Lagier et al., 2016, 2018).

Regardless of these two major techniques (culturomics and metagenomics), the processing and preparation of samples remain key factors to be considered before culture and sequencing.

Therefore, sampling and storage conditions, together with the time delay between the collection of the stool sample and its transport to the laboratory, affect the viability and the diversity of intestinal bacteria in the fecal flora (Moore et al., 1978; Bunthof and Abee, 2002; Cardona et al., 2012; Gorzelak et al., 2015; Nishimoto et al., 2016), and thus impacts the recovery of these microorganisms. Bacterial viability and survival have been challenging for many microbiologists, since the main target remains the culturing of all accessible microorganisms.

Most bacteria that colonize the human gut are anaerobic; they are 100–1000 times more numerous than aerobic bacteria (Loesche, 1969; Finegold, 1995). Anaerobic bacteria vary according to their sensitivity to oxygen and are often unable to survive in its presence (Rolfe et al., 1978). A recent study accurately measured the evolution of the oxygen level in the intestine and showed that it remains below 1 mmHg (Albenberg et al., 2014).

Traditionally, the quantification of human intestinal bacteria is performed by the plate count technique, which is considered the “gold standard” of bacterial quantification but remains time-consuming. Recently, alternative culture-independent methods have been used to achieve the enumeration of bacteria, such as flow cytometry (Davey, 2011; Vital et al., 2012; Zahavy et al., 2012), quantitative real-time PCR (Jervøe-Storm et al., 2005; Rezasoltani et al., 2017), FISH (Franks et al., 1998; Harmsen et al., 2000), electron microscopy and Gram staining (Hugon et al., 2013). However, many discrepancies were found between these techniques (Staley and Konopka, 1985).

Here, we used two quantification techniques to evaluate many culture conditions and sample conservation media by implementing new strategies to improve bacterial viability and conservation. To this end, we have designed three experimental protocols to study the effect of atmospheric oxygen on the viability of intestinal bacteria. We have proposed methods capable of improving the culture process, such as optimized culture conditions, along with a protectant medium that allowed for an in-depth study of the human gut microbiota. We also used a quantitative viability approach in which flow cytometry and serial plating helped in detecting bacterial viability and revealed important traits suggesting the end of the uncultured bacteria hypothesis.

## Materials and Methods

### Stool Samples Collection

Fresh stools were obtained from eight healthy donors (five men and three women) from Marseille, France. More detailed information is summarized in Supplementary Table 1.

None of the donors received antibiotics in the 3 months prior to sampling and did not suffer from any gastrointestinal tract manifestation. Volunteer donors were informed, and written consent was obtained, and the project received the ethics committee’s agreement under number 2016-011.

### Preparation of Stool Samples and Strategies to Target Fecal Microbial Cells

#### The Routinely Used Laboratory Protocol

In this protocol, all manipulations (mixing, filtration, serial dilutions and plating) were realized under a sterile hood. Briefly, stools were collected in a sterile stool container; right after sampling, a GasPak generator (Becton Dickinson, Sparks, MD, United States) was introduced into the container which was immediately closed, and kept in a plastic zippered pocket until it was reopened under a sterile hood and exposed to oxygen for 1 h and 30 min. 50 g of fecal matter was blenderized (BOSCH Ultracompact 400W) in 250 ml of normal saline solution (Fresenius Kabi, Sevres, France) for 5 min, followed by a filtration step using coffee strainers to remove big aggregates, such as undigested food or human cells. The slurry was centrifuged at 6000 × *g* for 15 min and re-suspended in a normal saline solution (Figure 1).

**FIGURE 1:** Schematic representation of the protocols used. The routine protocol (black arrows): the stool was exposed to oxygen for more than 1 h without any protectant medium. The optimized protocol (blue arrows): the stool was exposed to oxygen for more than 1 h and conserved in the protectant medium. The implemented optimized protocol (red arrows): the stool was exposed to oxygen less than 2 min, conserved in the protectant medium and all manipulations were performed inside the anaerobic chamber. The enumeration of bacterial cells was performed by Flow cytometry (FCM) and by the plate count method (CFU).

#### The Optimized Protocol Using a Protectant Medium for a Better Preservation and Survival of Cultured Bacteria

We used a protectant medium containing antioxidants patented under number N°1H53316 CAS 25 FR. The composition is detailed in Supplementary Table 2. Our medium proved its efficiency to preserve the gut bacteria, especially anaerobic bacteria, even after freezing and/or a freeze-drying process. We tested the viability of many anaerobic bacteria after freeze-drying in the presence and absence of the protectant medium (data not shown). Stools were then treated under the same conditions as the old routine protocol, except that the slurry was re-suspended in the protectant medium (Figure 1).

#### The Optimized Protocol Combining the Use of the Protectant Medium and Work Under an Anaerobic Chamber

Stools were collected in a sterile stool container containing 50 ml of the protectant medium. Stools were then treated under the same conditions as the old routine protocol, except that the container was opened in an anaerobic glove box (Don Whitley Scientific Limited, West Yorkshire, United Kingdom) with a gas mixture consisting of CO_2_, H_2_, N_2_ (15%; 5%; 80%). Finally, the slurry was re-suspended in the protectant medium (Figure 1).

### Enumeration of Bacteria Using the Culture-Dependent Method (CFU Counts) and Culture-Independent Method (Flow Cytometry Counts)

The enumeration of bacteria was performed using two methods; culture-dependent (CFU counts) and culture-independent (FCM). Serial dilutions from 10^–1^ to 10^–10^ were realized for the counting or enumeration. Dilutions were realized under both aerobic and anaerobic conditions, respectively, under a sterile hood, and under an anaerobic chamber.

### Culture: Plate Counting Method (CFU)

Regarding the culture plate counting method, serial dilutions ranging from 10^–1^ to 10^–10^ were performed on the stool samples suspended in phosphate buffered saline (PBS) (Life Technologies, Paiseley, United Kingdom). After homogenization, 10 μl of each dilution was spread onto Columbia sheep blood agar plates (BioMérieux, Marcy-l’Étoile, France) and then incubated at 37°C under anaerobic conditions using the GasPak^®^ system. It should be noted that we measured the oxygen level after putting on the Gaspak bag, which decreased from 1.3 to 1.4% after a few min and remained stable after 12 h of incubation. The colonies that appeared on plates were incubated for 48 h and counted. This process was carried out in triplicate.

For the routine and optimized protocols, plating was achieved 100–110 min after sampling under a sterile hood, and for the implemented optimized protocol, plating was performed in the anaerobic chamber 30 min after sampling and preparation of the sample. The rate of oxygen in the anaerobic chamber during the preparation of the samples and plating was of 0.3% O_2_.

### Enumeration by Flow Cytometry

We followed the principle of serial dilution and chose the best dilution for the optimal event rate for absolute enumeration. The LIVE/DEAD BacLight kit (Invitrogen, Eugene, United States) was used as proposed by the manufacturer. Live cells (untreated) and dead cells (isopropanol-treated) of different bacterial suspensions were used to adjust the flow cytometer as well as to optimize the dye ratio if necessary. After optimizing the dye concentration and the cytometer parameters for the detection, 1 ml of a diluted fecal sample at a 10^–3^ dilution (which was the best concentration for optimal flow rate and events counts) was stained with 1 μl of SYTO9 and 1 μl of PI, followed by an incubation for 15–20 min in the dark at room temperature. Then, beads (CytoCount, Dako) were added for quantification. As for flow cytometry, we used an LSR Fortessa (Becton Dickinson). Data acquisition was performed using log scales for instrument scatter parameters, forward scatter (FSC) and side scatter (SSC), respectively, associated with size and internal complexity of the event analyzed. Protocol threshold was adjusted on FSC parameter. Acquisition and analysis were performed using the “BD FACSDiva Software.” The number of collected events was fixed for all specimens. We used fluorescent beads, which are clearly distinguishable from fluorescent stained bacteria. The concentration of both live and dead bacteria was determined using the following equation:

(1) $$\frac{\mathrm{Number}\,\mathrm{of}\,\mathrm{cells}\,\mathrm{counted}}{\mathrm{Number}\,\mathrm{of}\,{\mathrm{CytoCount}}^{\mathrm{TM}}\,\mathrm{Beads}\,\mathrm{Counted}}\times {\mathrm{CytoCount}}^{\mathrm{TM}}\,\mathrm{Concentration}\times \mathrm{Dilution}\,\mathrm{Factor}$$

All the experiments and the staining steps were carried out under aerobic and anaerobic conditions and in triplicate for each stool sample. For anaerobic conditions, all staining procedures were performed under anaerobic conditions, except for the acquisition process on the flow cytometer, which was carried out under aerobic conditions.

### Statistical Analysis

Statistical analysis was performed using the Mann–Whitney *t*-test to identify statistically significant differences between different protocols (Prism v5.0, GraphPad). Descriptive statistics were calculated and reported as means and standard deviations. A *P* < 0.05 was considered statistically significant.

## Results

### Results of the Quantification of Bacteria Using CFU Counts and Flow Cytometry

#### Aerobic Conditions: The Routine and the Optimized Protocols

Some of the stool samples were processed twice. The 13 stool samples collected from eight donors were exposed to air for more than 1 h, with normal saline solution in the routine protocol and with the protectant medium in the optimized protocol. The total number of bacterial cells and the percentages of cultured bacteria determined by agar plating and FCM are shown in Table 1.

**TABLE 1:** The routine and the optimized protocol.

**Samples**	**Protocols**	**Flow cytometry (10^9^ cell/ml)**				**Cultured bacteria (10^9^ CFU/ml)**		
		**Total**	**Live**	**Dead**	**Injured**	**Total**	**Anaerobe**	**Aerobe**
1	Routine	10.64	6.39	3.84	0.41	3.53	3.00	0.53
	Optimized	11.15	7.08	3.76	0.31	6.53	6.00	0.53
2	Routine	6.30	3.90	1.80	0.60	2.70	2.00	0.70
	Optimized	9.64	6.59	2.41	0.64	5.70	5.00	0.70
3	Routine	10.38	6.92	2.73	0.73	2.10	2.00	0.10
	Optimized	12.11	7.80	2.98	1.33	4.12	4.10	0.02
4	Routine	11.08	5.91	3.66	1.51	3.67	3.60	0.07
	Optimized	12.71	7.25	3.89	1.57	6.04	6.00	0.04
5	Routine	5.63	3.88	1.20	0.55	1.90	1.20	0.70
	Optimized	9.27	6.80	1.60	0.87	3.26	2.46	0.80
6	Routine	12.72	6.29	3.82	2.61	2.16	2.00	0.16
	Optimized	12.16	6.86	3.34	1.96	3.20	3.00	0.20
7	Routine	8.66	6.05	1.91	0.70	2.22	2.20	0.02
	Optimized	11.15	6.43	2.40	2.32	2.97	2.90	0.07
8	Routine	4.58	3.42	1.00	0.17	1.10	1.00	0.10
	Optimized	5.52	4.82	0.48	0.22	2.40	2.30	0.10
9	Routine	6.51	1.62	4.34	0.55	1.02	1.00	0.02
	Optimized	8.27	2.40	5.15	0.72	1.83	1.76	0.07
10	Routine	7.46	4.03	3.13	0.30	2.41	2.40	0.01
	Optimized	8.82	4.99	3.48	0.35	4.44	4.38	0.06
11	Routine	11.15	4.44	5.63	1.08	3.01	3.00	0.01
	Optimized	11.57	5.26	4.67	1.64	4.03	3.50	0.53
12	Routine	8.03	3.63	3.37	1.03	2.42	2.22	0.20
	Optimized	10.31	4.62	4.67	1.03	3.56	3.33	0.23
13	Routine	6.33	3.37	1.85	1.12	2.20	1.50	0.70
	Optimized	6.70	3.80	1.97	0.93	2.44	2.00	0.44
Mean	Routine	8.42(±2.54)	4.60(±1.56)	2.94(±1.35)	0.87(±0.64)	2.34(±0.78)	2.08(±0.79)	0.25(±0.28)
	Optimized	9.95(±2.19)	5.74(±1.57)	3.14(±1.34)	1.07(±0.65)	3.88(±1.46)	3.59(±1.42)	0.29(±0.27)

*Total cell counts and total cultured anaerobes and aerobes from 13 samples performed by FCM and by CFU counts.*

The FCM results showed a total cell count that ranged from 4.58 × 10^9^ to 1.27 × 10^10^ cells/ml for the 13 samples treated only with normal saline solution in the routine protocol, while it was between 5.52 × 10^9^ and 1.27 × 10^10^ cells/ml for samples treated with a protectant medium in the optimized protocol (Table 1). The mean percentage for each population is presented in Figure 2. In the routine protocol, only 55.52% (±13.78%) of the cells were live, 34.58% (±13.07%) were dead and around 9.90% (±5.15%) were injured. However, in the optimized protocol, 58.51% (±14.28%) were live, 31.21% (±13.58%) were dead and 10.28% (±5.24%) were injured.

**FIGURE 2:** Total cell counts by Flow cytometry (FCM) (dead, live and injured bacteria) and Colony forming unit (CFU) counts (aerobes and anaerobes bacteria) in the three protocols. The percentage of culturability was counted from total cells in fecal samples and from live cells counted by FCM. Significant differences between protocols were highlighted using the Mann–Whitney’s test.

The percentages of culturability were calculated from total living bacteria counted by FCM.

In the routine protocol, only 28.24% (±6.89%) were culturable from 55.52 % (±13.78%) viable bacteria. In the optimized protocol, 39.55% (±13.28%) were culturable from 58.51% (±14.28%) viable bacteria (Figure 2). Thus, the majority of cultured bacteria was anaerobic, and they were 100 times more numerous than aerobic bacteria (Figure 2).

The mean percentage of cultured cells counted using the CFU technique and the viable cells counted by FCM are heterogeneous for the 13 samples of the two protocols. In the routine protocol, counts were at 4.6 × 10^9^ cell/ml (FCM) versus a total of 2.34 × 10^9^ CFU/ml. Among the 2.34 × 10^9^ CFU/ml count, 2.09 × 10^9^ CFU/ml was anaerobic and 2.6 × 10^8^ CFU/ml was aerobic. However, in the optimized protocol, we obtained 5.74 × 10^9^ cell/ml (FCM) versus a total of 3.88 × 10^9^ CFU/ml; 3.59 × 10^9^ CFU/ml was anaerobic and 2.91 × 10^8^ CFU/ml was aerobic.

The cultured bacteria counted by the CFU method were half as numerous as those counted by the FCM method. The rate was much lower for samples dissolved in a normal saline solution in the routine protocol compared to those of the optimized protocol in the presence of the protectant medium. The count was statistically significant for both protocols; the routine protocol had a *P* of 0.005 (Figure 3A) and the optimized protocol had a *P* of 0.006 (Figure 3B).

**FIGURE 3:** **(A)** Routine protocol, **(B)** optimized protocol versus **(C)** implemented optimized protocol. The graphs represent Mann–Whitney’s test performed to assess the significance of the number of viable colonies measured by the CFU method and FCM.

#### Anaerobic Manipulations: The Implemented Optimized Protocol

Five stool samples were tested using the implemented optimized protocol, all manipulations were realized under anaerobic conditions and exposure to oxygen did not exceed 2 min. The total number of cells and cultured bacteria tested according to the optimized protocol used is shown in Table 2.

**TABLE 2:** The implemented optimized protocol.

**Samples**	**Protocols**	**Flow cytometry (10^9^ cell/ml)**				**Cultured bacteria (10^9^ CFU/ml)**		
		**Total**	**Live**	**Dead**	**Injured**	**Total**	**Anaerobe**	**Aerobe**
1	Optimized	11.94	7.65	3.02	1.27	6.89	6.87	0.02
2	Optimized	9.77	6.06	3.00	0.71	5.06	5.00	0.06
3	Optimized	11.52	6.87	2.87	1.79	6.30	6.20	0.10
4	Optimized	9.62	6.40	2.12	1.10	5.72	5.35	0.37
5	Optimized	10.56	5.94	2.70	1.92	4.87	4.50	0.37
Mean	Optimized	10.68(±1.03)	6.58(±0.69)	2.74(±0.37)	1.35(±0.49)	5.76(±0.84)	5.58(±0.94)	0.18(±0.17)

*Total cell counts and total number of cultured anaerobes and aerobes from five samples performed by FCM and by CFU counts.*

Total cell count ranged between 9.62 × 10^9^ and 1.19 × 10^10^ for the five samples used, and the mean percentages of bacterial cell counts of live, injured and dead bacteria were respectively 61.69% (±3.98%), 25.70% (±3.14%), and 12.61% (±4.28%) (Figure 2). Regarding the CFU method, the mean percentages of cultured bacteria in the implemented optimized protocol were 54.00% (±4.84%) from 61.69% (±3.98%) live bacteria (Figure 2).

Under anaerobic conditions, the mean percentage of live cells counted by FCM did not differ significantly from the cultured cell count (CFU; *P* = 0.222; Figure 3C). It was 6.58 × 10^9^ cell/ml (FCM) versus a total of 5.76 × 10^9^ CFU/ml; 5.58 × 10^9^ CFU/ml was anaerobic and 1.82 × 10^8^ CFU/ml was aerobic (Figure 2).

## Discussion

The main objective of this study was to evaluate the conservation of bacteria in fresh fecal material. Two methods were used and optimized to compare the bacterial viability and culturability under three different conservation conditions.

We observed that anaerobes outnumbered aerobes by 1–2 logs, thus the total bacterial cell count varied between fecal samples (Tables 1, 2), regardless of the counting method (FCM or CFU) or the processing conditions. These differences can be due to many factors and are donor-dependent (nutrition, diet, lifestyle…etc.) (Clemente et al., 2012; Conlon and Bird, 2014).

Our results showed that the most represented population in the fresh fecal samples was the live microbial population, regardless of the sample conditioning. We found 55.52% in the routine protocol, 58.51% in the optimized protocol and 61.69% in the implemented optimized protocol, while dead cells were 34.58, 31.21, and 25.70%, respectively. The implemented optimized protocol gave us the highest percentage of viability (∼62%) and the lowest fraction of dead bacteria (∼26%). The study by Apajalahti et al. (2003) showed approximately the same results, except that they only detected dead bacteria (IP-staining) and found a mean of 28% for the dead microbial population ranging from 17 to 34%. In addition, our implemented optimized protocol showed a higher percentage of viable cells (∼62%), compared to the study reported by Ben-Amor et al. (2005), where 49% were live, 32% were dead and 19% were injured, which is higher than our results under the same anaerobic conditions (25.69% dead and 12.60% injured).

Regarding culturability, samples without any protectant medium that were exposed to oxygen for 90 min allowed us to culture 50.86% of total living cells (routine protocol), while the percentage of culturability increased to 67.59% in the presence of our protectant medium (the optimized protocol) containing antioxidants (N°1H53316 CAS 25 FR). Interestingly, the culturability increased to 87.53% when sampling, collection and sample preparation were performed in an oxygen-free atmosphere (the implemented optimized protocol). We gained viability and culturability for all samples in our implemented optimized protocol. This protocol conserved the samples and the bacterial community for a better yield and isolation rates.

In the literature, the percentage of cultivability of gut bacteria varies from one study to another (10–93%). These differences can be explained by the use of different counting techniques, culture conditions and media used (Macfarlane and Gibson, 1994; Langendijk et al., 1995; Wilson and Blitchington, 1996). Moore’s study showed that only 63.75% of microscopic counts were cultivated when the delay between sampling and sending the samples to the laboratory was 2 h (Moore and Holdeman, 1974b). They suggested that the difference was probably related to the exposure of specimens to oxygen without any protection before processing. In another study, they demonstrated that a mean of 93% of viable cells counted by microscopy could be cultivated when appropriate techniques were employed, such as using special media and anaerobic conditions (Moore and Holdeman, 1974a).

In our study, we showed that the delay between sample collection and sample processing was very important and should be as short as possible (<2 min). Several studies reported a low percentage of culturability when the delay between sampling and processing was more than 1 h without any protection. Different rates of culturability were found depending on the delay. For instance, scientists cultured in different studies 37% of bacteria from total microscopic counts (Langendijk et al., 1995), while 15% (Langendijk et al., 1995), 14% (Welling et al., 1997), 54% (Matsuki et al., 2002), and 30% (Franks et al., 1998) were cultured from the total cells counted by DAPI staining. The study conducted by Leonardo and colleagues showed that the highest counts of cultured anaerobic bacteria were obtained when the time between sample collection and sample processing in the anaerobic chamber was less than 15 min and decreased by 1–3 logs after 2 h (Mata et al., 1969). Another study by Brusa et al. (1989) reports the exposure of 10 strict anaerobic bacteria to oxygen for variable durations: after 4–5 min, the percentage of viable bacterial cells was 50%, dropping to 0.1% after 40 min and no cell survived after 2 h.

A possible reason that a greater proportion of the bacterial community was not cultured when the fresh sample was exposed to O_2_ might be the fact that oxygen-sensitive cells were in the viable but non-culturable state, or either injured or dead. Loesche (1969) determined two classes of anaerobic species regarding their tolerance to oxygen; “moderate anaerobes” were capable of growing at 2–8% oxygen levels and were exposed to room atmosphere for 90 min, and “strict anaerobes” were unable to grow in an atmosphere containing more than 0.5% of oxygen.

## Conclusion

Our current work has confirmed the importance of sample conditioning and processing to obtain the best culture conditions and isolation rates. We proposed a great conditioning medium capable of preserving the bacterial viability in the samples. Our work contributes to the culturomics field by reducing the exposure to oxygen between sample collection and sample processing.

A complementary metagenomic study is ongoing to compare the metagenomic data of the 3 FACS fractions of live, dead and injured bacteria in human feces to the data of the bacteria cultured in the same samples using different culturomics approaches. This will help clarifying whether the majority of uncultured bacteria were dead or live. It may also help in defining what is uncultured, due to their need for optimal culture conditions.

By using two methods of quantification under aerobic and anaerobic conditions, our results highlight the need to optimize collection procedures and storage conditions. This objective can be achieved using rigorous and controlled anaerobic methods, especially during the sampling and throughout the culturomics process. The comprehension of this concept is essential for the development of optimal techniques for isolating new and fastidious anaerobic bacteria and studying the role of these microorganisms in human health.

## Data Availability

All datasets generated or analyzed for this study are included in the manuscript and/or the Supplementary Material.

## Ethics Statement

This study was reviewed and approved by the IHU Méditerranée Infection ethics committee (Approval Number: 2016-011). Written informed consent was obtained from all participants.

## Author Contributions

SB performed the experiments and wrote the manuscript. J-CL reviewed the drafts of the manuscript. SB and JBK performed the flow cytometry analysis. JBK drafted the flow cytometry section. JBK and DR were responsible for the data interpretation and critically revised the manuscript. All authors contributed to the revised version of the manuscript, and read and approved the final version of the manuscript.

## Conflict of Interest Statement

The authors declare that the research was conducted in the absence of any commercial or financial relationships that could be construed as a potential conflict of interest.
